# Whole Transcriptomic Analysis of Key Genes and Signaling Pathways in Endogenous ARDS

**DOI:** 10.1155/2022/1614208

**Published:** 2022-10-04

**Authors:** Yongpeng Xie, Jiye Luo, Wenxia Hu, Chongchong Ye, Panpan Ren, Yanli Wang, Xiaomin Li

**Affiliations:** ^1^Department of Emergency and Critical Care Medicine, Lianyungang Clinical College of Nanjing Medical University, The First People's Hospital of Lianyungang, China; ^2^The Institute of Emergency Medicine of Lianyungang, Lianyungang City, Jiangsu Province, China 222000

## Abstract

**Objective:**

To analyze the differentially expressed genes (DEGs) in rats with endogenous acute respiratory distress syndrome (ARDS) lung injury and explore the pathogenesis and early diagnostic molecular markers using whole transcriptomic data.

**Methods:**

Twelve 8-week-old male Sprague Dawley rats were selected and randomly and equally divided into ARDS lung injury group and normal control group. RNA was extracted from the left lung tissues of both the groups and sequenced using the paired-end sequencing mode of the Illumina Hiseq sequencing platform. The DEGs of miRNA, cirRNA, lncRNA, and mRNA were screened using DESeq2 software, and the ceRNA regulatory network was constructed using Cytoscape. Gene ontology (GO) and Kyoto Encyclopedia of Genes and Genomes (KEGG) enrichment analysis were performed using the mRNA DEGs. STRING and Cytoscape software were used to construct the protein interaction network and identify the 15 key genes, which were verified using quantitative real-time polymerase chain reaction (qRT-PCR).

**Results:**

Based on different screening conditions, and compared with the control group, the ARDS lung injury group showed 836 mRNA DEGs (386 upregulated and 450 downregulated), 110 lncRNA DEGs (53 upregulated and 57 downregulated), 19 circRNA DEGs (3 upregulated and 16 downregulated), and 6 miRNA DEGs (5 upregulated and 1 downregulated gene). GO showed that the DEGs of mRNA were mainly involved in biological processes, such as defense response to lipopolysaccharide and other organisms, leukocyte chemotaxis, neutrophil chemotaxis, and cytokine-mediated signaling. KEGG enrichment analysis showed that the DEGs played their biological roles mainly by participating in IL-17, TNF, and chemokine signaling pathways. The PPI analysis showed a total of 281 node proteins and 634 interaction edges. The top 15 key genes, which were screened, included *Cxcl10*, *Mx1*, *Irf7*, *Isg15*, *Ifit3*, *Ifit2*, *Rsad2*, *Ifi47*, *Oasl*, *Dhx58*, *Usp18*, *Cmpk2*, *Herc6*, *Ifit1*, and *Gbp4*. The ceRNA network analysis showed 69 nodes and 73 correlation pairs, where the key gene nodes were miR-21-3p, Camk2g, and Stx2.

**Conclusions:**

The chemotaxis, migration, and degranulation of inflammatory cells, cytokine immune response, autophagy, and apoptosis have significant biological functions in the occurrence and development of endogenous acute lung injury during ARDS. Thus, the camk2g/miR-21-3p/lncRNA/circRNA network, CXCL10/CXCR3, and IL-17 signaling pathways might provide novel insights and targets for further studying the lung injury mechanism and clinical treatment.

## 1. Introduction

Acute respiratory distress syndrome (ARDS) is a common acute and critical illness in the field of critical care medicine [1]. An international epidemiological LUNG SAFE study showed that the incidence of ARDS among the intensive care unit (ICU) patients was about 10% [2]. In recent years, severe acute respiratory infections, which endanger human health, have been frequently occurring, such as severe acute respiratory syndromes (SARS) in 2003 [3], influenza A (H1N1) in 2009, and novel coronavirus pneumonia (corona virus disease-19 (COVID-19); the latter is still spreading around the world) [4]. Most critically ill patients progress to ARDS, having a fatality rate of over 40% [5]. Although significant advancements have been made in understanding and treating the pathophysiology of ARDS in the past 20 years, the underlying mechanism of acute lung injury in endogenous ARDS is not yet fully understood. Furthermore, specific biomarkers and effective therapeutic targets are lacking [6]. RNA-sequencing (RNA-Seq) is a recently developed high-throughput sequencing technology, which has the advantages of rapid analysis and high resolution. In the present study, RNA-Seq technology was used to study the expression profiles of lung injury genes in the endogenous subtype of lipopolysaccharide (LPS)-induced ARDS, and the key genes and pathways were screened. The purpose of this study was to provide novel ideas for studying the mechanism of endogenous ARDS lung injury and to explore therapeutic targets and specific biomarkers.

## 2. Materials and Methods

### 2.1. Experimental Animals and Groups

This study was approved by the Medical Ethics Committee of Lianyungang Clinical College of Nanjing Medical University, and all the animal experiments were performed strictly according to the requirements of animal ethics (Number: KY20200311001, Date: March 11, 2020). A total of 12 healthy clean-grade male Sprague Dawley rats were selected. Rats were 6-8 weeks old, weighing 230-250 grams each. Rats were divided randomly into blank control group (N group) and experimental group (LPS group) with 6 animals in each group. The endogenous ARDS lung injury rat models (LPS group) were established by instilling LPS (Sigma-Aldrich, St. Louis, MO, USA; 10 mg/kg) into their airways.

### 2.2. Pathological Observation of Lung Tissues

After 36 h, rats were anesthetized by an intraperitoneal injection of xylazine (Sigma-Aldrich, St. Louis, MO, USA; 8 mg/kg) and ketamine (Hengrui, China; 80 mg/kg). After successful anesthetization, the rats were sacrificed by cardiac puncturing and bloodletting, and the sample specimens were collected for examination. The wet/dry weight ratio of the middle lobe of the right lung tissue was calculated to determine the severity of pulmonary inflammatory infiltration and edema. In brief, the lung tissues of the right upper lobe of the rats were collected, dehydrated with gradient alcohol, embedded in paraffin, and sectioned. Damage to the lung tissue was observed at low, medium, and high magnification using an Olympus microscope.

### 2.3. Total RNA Extraction from Lung Tissues

The total RNA was extracted from the lung tissues using RNA extraction kits (Thermo Fischer Scientific, Waltham, MA, USA). The purity and RNA integrity factor of the extracted RNA samples were detected using Thermo Nanodrop one ultra-micro spectrophotometer and Agilent2100 bioanalyzer (Santa Clara, CA, USA), respectively, in order to meet the requirements of subsequent sequencing quality.

### 2.4. Sequence Preprocessing and Classification Annotation

In this study, the paired-end sequencing mode of the Illumina HiSeq sequencing platform was used for the high-throughput sequencing of multiple samples. Skewer software (v0.2.2) was used to dynamically remove the adapter sequence and low-quality fragments from the 3′ end of the sequencing reads. FastQC software (v0.11.5) was used to perform the preprocessing data quality control analysis. For each sample, STAR software (2.5.3a) was used to align the preprocessed sequencing reads with the reference genome sequences of the sequenced species, and RSEQC (v2.6.4) was used for the comparison statistical analysis. The sequence data after alignment and filtration was submitted to the Rfam database, RepBase sequence database, and miRBase database for the prediction analysis of new miRNAs, alignment annotation analysis of known miRNAs, and quantitative analysis of miRNAs, respectively. For transcripts assembled by StringTie (v1.3.1c), the assembled transcripts were classified by comparing the results of gff compared with the reference genome location information of known genes. The transcripts with o, i, x, j, and u and those with lengths greater than 200 bp and the number of exons ≥2 were retained for further screening. The partial transcripts with the potential of protein coding were removed using software system platforms, such as PLEK (1.2), CNCI (1.2.2), and Pfam. Long noncoding RNA (lncRNA) sequences obtained from the sequencing of samples were compared with the known lncRNA sequences using the blastn software platform. Known lncRNA sequences were then quantitatively analyzed. For the STAR alignment results, CIRCexplorer2 software (2.2.6) was used for predicting the front and rear positions of circular RNAs (circRNAs). The annotation and gene structure analysis of circRNA-derived genes were performed based on the location information of circRNA chromosomes.

### 2.5. Gene Expression Levels and Function Analysis

The mRNA expression levels were calculated using FPKM method, which refers to the number of fragments per kilobase in length from a protein-coding gene per million fragments. Quantitative calculations of miRNA and lncRNA were performed by the number of transcripts per million the number of fragments per kilobase length per million fragments from a transcript, respectively. The quantitative calculation of circRNA was performed by the number of transcripts per million spliced. The differentially expressed genes (DEGs) were screened out using DESeq software, followed by statistical analysis and visualization using software R (version 3.6.3), and visualized using volcano plots and heat maps for observing the differences in gene expression levels between the two groups. Gene ontology (GO) function enrichment analysis and Kyoto Encyclopedia of Genes and Genomes (KEGG) pathway enrichment analysis of the DEGs were performed for the functional annotation and classification. The mRNA expression profile dataset GSE32707 was downloaded from GEO (http://www.ncbi.nlm.nih.gov/geo/). This dataset includes mRNA expression data of 33 ARDS and 34 control samples (without sepsis or ARDS). Total RNA was extracted from the whole blood samples, and microarrays were prepared to determine the DEGs with screening conditions of |log2FC| ≥ 1 and *P* value < 0.05. A Venn diagram was drawn to identify the co-expressed DEGs in the two datasets (human DEGs and rat DEGs). Co-expressed DEGs were imported to the online STRING database for protein-protein interaction (PPI) analysis. Proteins with a comprehensive score of >0.7 in the PPI network graph were considered statistically significant. Cytoscape (version 3.9.1) plug-in cytoHubba was used to identify the top 15 most significant genes.

### 2.6. Construction and Analysis of mRNA-miRNA-lncRNA-circRNA Network

Whole transcriptome sequencing results, including those of miRNA, lncRNA, circRNA, and mRNA sequence information, were obtained and the base sequences were used to predict the miRNA-target relationship pairs. miRanda (v3.3a) was used to predict the target recognition sites of miRNA in the genome sequence. The threshold parameters used for this process are *S* > 150 and Δ*G* < −20 kcal/mol, where *S* is referred to the single residue-pair match scores and Δ*G* is the free energy for duplex formation. According to the expression levels of miRNAs and their predicted targets, including lncRNA, circRNA, and mRNA, Pearson's correlation coefficients associated with miRNA-predicted target correlation pairs were calculated. Pairs, which were significantly negatively correlated with regulating the expression of the miRNA-targets, were screened out. When the correlation coefficient of expression was >0.05 and the absolute value of Pearson's correlation coefficient was less than 0.7, the correlational possibility was excluded. These base sequences and predictions of expressions were summarized for subsequent competing endogenous RNA (ceRNA) prediction analysis. According to the screening results, the miRNA-target, miRNA-cirRNA, and mRNA-lncRNA (only DEGs) were identified and integrated. The obtained ceRNA relationship pairs were presented in the form of lncRNA/circRNA-microRNA-mRNA network.

### 2.7. RNA Extraction and Quantitative Real-Time Polymerase Chain Reaction (qRT-PCR)

The top 15 most significant genes were selected for verification using qRT-PCR (ABI 7500, Thermo Fischer Scientific, Waltham, MA, USA). Blood samples (PBMCs) from 20 patients with pulmonary endogenous ARDS and 10 age-matching healthy controls were collected. Total RNA was extracted from the samples using RNA extraction kits (Omega, Guangzhou, China). Reverse transcription of mRNA was performed using the Primescript RT main mixing kit (Takara, Dalian, China) for obtaining the corresponding cDNA. The amplification of the selected genes was performed using Ultra Sybr Mixture. Using the glyceraldehyde-3-phosphate dehydrogenase (*GAPDH*) gene as internal control, the mRNA expression levels of the top 15 key genes were detected. The PCR reaction conditions were as follows: initial denaturation at 95 °C for 10 min, followed by 45 cycles of denaturation at 95 °C 15 s, and annealing and elongation at 60 °C for 60 s. The experimental results were obtained as CT values, and the relative expression of mRNA was calculated using the 2^-*ΔΔ*CT^ method. Primer sequences for each gene are listed in Table 1.

## 3. Results

### 3.1. Pathological Damage during Endogenous ARDS Lung Injury

After 36 h of establishing the rat ARDS models, morphological observation and evaluation showed that the lungs of rats in the LPS group had signs of atelectasis, enlargement, and congestion; some even had edema fluid filled with endotracheal intubation. The wet/dry weight ratio of the lung tissue in the LPS group was significantly higher than that in the control group (5.263 ± 0.531 vs 4.325 ± 0.223) (*P* < 0.01). These findings reflected the permeability of the pulmonary blood vessels and indicated the severity of pulmonary inflammatory infiltration and edema. In the LPS group, the rat lung tissues showed more serious pathological damages, which were manifested as diffused alveolar damage, intra-plasmic congestion and edema, inflammatory cell infiltration, atelectasis, hyaline membrane formation, etc. (Figures 1(a) and 1(b)). In the control group, the alveolar walls were very thin, and most the alveoli did not contain any cells when observed by light microscope (Figures 1(c) and 1(d)).

### 3.2. RNA Extraction of Lung Tissue and Quality Control

The total amount of RNA extracted from the two groups was >0.2 *μ*g with a mass-volume concentration of >20.0 ng/*μ*L. Extracted RNA was of high purity and had good integrity, which met the standards of library construction. As shown in Figures 2(a) and 2(c), the quality, distribution, and homogeneity of the samples were sufficient, thereby meeting the standards of library construction. To evaluate the repeatability of the data within group, principal component analysis (PCA) was performed to observe similarities between the samples by reducing the dimension. As shown in Figure 2(b), blue circles represent rats in the control group, and red circles represent rats in the LPS group. Dots represent rats in the LPS group. The closer the sample distance, the closer the trend of gene expression in the samples. Together, the results showed good reproducibility of the RNA whole transcriptomic data of the two groups.

### 3.3. Identification of DEGs

A total of 2524 mRNA DGEs were identified between the two groups. With the screening conditions of |log2FC| ≥ 2 and *P* value < 0.01, the LPS group had 836 DEGs when compared to the control group, including 386 upregulated genes and 450 downregulated genes. The total number of lncRNA DEGs between the two groups was 4065, which was reduced to 110 after selected screening conditions, including 53 upregulated genes and 57 downregulated genes. The total number of circRNAs was 17,679, among which, only 19 circRNAs met the threshold of screening conditions and included 3 upregulated genes and 16 downregulated genes. The total number of miRNAs was 572, among which, 6 miRNAs met the thresholds of screening conditions and included 5 upregulated and 1 downregulated gene. The volcano plots of DEGs are presented in Figures 3(a)–3(d). After analyzing the DEGs of lncRNAs and mRNAs using R software, the top 40 DEGs of lncRNAs and mRNAs were visualized in heatmaps (Figures 3(e) and 3(f)).

### 3.4. GO/KEGG Enrichment Analysis and Gene Set Enrichment Analysis (GSEA) Analysis

The GO function and KEGG pathways enrichment of the 836 DEGs were analyzed. Using the conditions of *P*_adj_ < 0.01 and *q* value < 0.2, there were 577 biological processes (BPs), 32 cellular components (CCs), and 52 molecular functions (MFs). The BPs of DEGs mainly included the response to LPS, defense response to other organisms, leukocyte chemotaxis, neutrophil chemotaxis, and cytokine-mediated signaling pathways. Among the CCs, DEGs were mainly enriched in ion channel complexes, transmembrane transporter complexes, transport complexes, and extracellular matrix. For MFs, the DEGs were significantly enriched in cytokine activity, chemokine activity, receptor modulation activity, and cytokine receptor binding (Table 2). KEGG pathway enrichment analysis showed that a total of 33 signaling pathways were significantly enriched in the LPS group. DEGs were significantly involved in cytokine-cytokine receptor interaction and interleukin-17 (IL-17), tumor necrosis factor (TNF), nuclear factor kappa-B (NF-*κ*B), and chemokine signaling pathways. GSEA was performed to identify the possible underlying mechanism of the lung injury process in ARDS. The results showed that the set of genes involved in autophagous and apoptotic activities had a significant positive correlation with the lung injury process in ARDS (Figures 4(a) and 4(b)).

### 3.5. PPI Analysis and ceRNA Network Construction

The mRNA expression dataset GSE32707 was downloaded from GEO (http://www.ncbi.nlm.nih.gov/geo/). Using the |log2FC| ≥ 1 and *P* value < 0.05 as screening conditions, 449 human DEGs were selected. In the rat mRNA expression datasets, the screening conditions resulted in a total of 2524 DEGs. A Venn diagram was used to identify the co-expressed DEGs in the two datasets (Figure 5(b)). The 130 co-expressed DEGs were imported into the online STRING database for PPI network analysis (https://cn.string-db.org), which is shown in Figure 5(a). The PPI network analysis showed a total of 130 node proteins with 419 interacting edges (the expected number of edges was 140), 6.45 average node degree, 0.432 average local clustering coefficient, and <1.0e-16 enrichment *P* value. This meant that the proteins had more interactions among themselves than the expected interactions among a random set of proteins of the same size and degree distribution. This enrichment indicated that the differential proteome might be involved in a biological activity as a group during ARDS lung injury or was at least partially biologically connected.The top 15 key proteins including hematopoietic cell kinase (HCK), fetal growth restriction (FGR), S100A9, cytochrome b-245 beta chain (CYBB), salmonella pathogenicity island 1 (SPI1), CD14, chemokine C-X-C ligand 10 (CXCL10), formyl peptide receptor 1 (FPR1), Fc receptor gamma (FCER1G), colony-stimulating factor receptor (CSF3R), G protein-coupled receptor1 (CXCR1), Fc fragment of IgG receptor 1a (FCGR1A), Aquaporin 9 (AQP9), rac family small GTPase 2 (RAC2), and signal transducer and activator of transcription 3 (STAT3) were screened out using Cytoscape plug-in cytoHubba with degree value >10 (Figure 5(c)). Furthermore, ceRNA analysis showed that miRNA target genes were comprehensively predicted using the two-part computational prediction steps, including miRNA-cirRNA sequence matching and evaluating the calculation of energy stability. This resulted in a total of 2 circRNAs, 1 miRNA miR-21-3p, and 3 miRNA-circRNAs. According to the differential miRNA, RNAInter (http://www.rna-society.org/raid/) was used to predict the lncRNAs regulated by the rat miRNA miR-21-3p, which showed that there was no lncRNA regulation by this miRNA. Target prediction of differentially expressed miRNAs was performed using miRanda to obtain the differential mRNAs regulated by rno-miR-21-3p. According to the distance between the lncRNA and known protein-coding gene, the target prediction was set to 100 kb upstream and downstream of the lncRNA in order to obtain the differential lncRNA-mRNA targets, integrated miRNA-target, miRNA-cirRNA, and mRNA-lncRNA (only DEGs). We then constructed an mRNA-miRNA-lncRNA-circRNA regulatory network (ceRNA network) containing 69 nodes and 73 relational pairs as shown in Figure 5(d); the green circles are downregulated mRNAs, the red triangles are upregulated miRNAs, the blue diamonds are downregulated known lncRNAs, the gray diamonds are downregulated predicted lncRNAs, and the orange hexagons are circRNAs. Key nodes were miR-21-3p, calcium ion/calmodulin-dependent protein kinase II gamma (Camk2g), and Shiga toxin 2 (Stx2).

### 3.6. qRT-PCR Validation Analysis

The top 15 key genes, which were screened using Cytoscape plug-in cytoHubba, were selected as representative target genes for validation using qRT-PCR analysis. The relative expression of these genes in the 6 LPS groups and normal samples is shown in Figure 6(a). Following the analysis of GSE32707 dataset using R software, the expression of selected genes in the LPS and normal groups are shown as box plots (Figure 6(b)). To verify the RNA-Seq results, DEGs were validated in 20 ARDS patients and 10 control groups using qRT-PCR. The results showed that the changing trend of 7 key genes (*CYBB*, *CD14*, *CXCL10*, *FCER1G*, *CXCR1*, *FCGR1A*, and *STAT3*) was consistent with the RNA-Seq results (all *P* < 0.05). No statistically significant differences were observed in other 8 genes (Figure 6(c)).

## 4. Discussion

Defining the homogeneous subgroups in critical illness syndromes, such as ARDS, is a current research focus in the field of acute and critical clinical care [7]. It has also been gradually discovered that there are large differences between the clinical characteristics (phenotype) or molecular mechanism-related responses to treatment (endogenous type) and/or prognostic risk (prognosis) among critically ill subgroups [8]. Clinical studies have shown that patients with the pulmonary endogenous ARDS phenotype are more ill compared to those with exogenous pulmonary ARDS, which is reflected by their poorer recovery from lung injury, lower success rate of extubation, higher short-term mortality, and possibly worse long-term prognosis [9, 10]. However, despite the focus of many studies on this, the complex and diverse mechanism of endogenous lung injury is not yet fully understood, and the relatively effective treatment methods and early diagnostic biomarkers are also lacking [11]. Based on the current situations, the present study explored the key genes and signaling pathways involved in the pathogenesis of endogenous lung ARDS, which is a special but common subtype of lung injury, using the whole transcriptomic data and explored the mechanism of lung injury, as well as provided insights into the prevention and treatment targets.

In this study, a rat model of ARDS lung injury was established by instilling LPS into their airways, and ARDS was determined according to respiratory distress symptoms, the oxygenation index, and pulmonary pathological changes in rats [12]. Rat models of ARDS were fully in line with the common clinical conditions and pathological changes of the patients with endogenous ARDS lung injury. Lung tissue of the LPS (ARDS) group showed severe pathological damage, which was mainly manifested as diffused alveolar damage, including congestion and edema in the alveoli and interstitium, atelectasis, and hyaline membrane formation. There was also a significant infiltration of inflammatory cells around the alveoli, bronchi, and especially the pulmonary arterioles. To the best of our knowledge, this is the first analysis integrating mRNA, lncRNA, circRNA, and miRNA profiles in endogenous ARDS. Moreover, a total of 836 mRNAs, 110 lncRNAs, 19 circRNAs, and 6 miRNAs were identified from the endogenous ARDS injury lung.

The GO/KEGG functional enrichment analysis of whole transcriptomic data from endogenous ARDS lung tissue revealed that the DEGs were enriched in many BPs, including defensive responses to lipopolysaccharide-induced, leukocyte chemotaxis, neutrophil chemotaxis, and cytokine-mediated signaling pathways. DEGs showed chemokine activity through transcriptional proteins and binding to chemokine receptors, thereby further mediating the invasion and infiltration of inflammatory cells in alveoli, peribronchioles, pulmonary arteries, and pulmonary capillaries. This causes inflammatory cells to release inflammatory factors through autocrine, paracrine, and degranulation processes and exert receptor regulatory activity and receptor-ligand activity for mediating inflammatory cascade responses [13]. These responses result in damaged alveolar epithelial cells and changes in pulmonary capillary permeability, further causing refractory pulmonary edema, atelectasis, refractory hypoxemia, and respiratory distress symptoms [14, 15]. Many inflammatory cells infiltrate around the pulmonary arterioles, resulting in the vascular smooth muscle cell edema, inflammatory proliferation of fibrous connective tissue, and severe hypoxemia, which mediate acute pulmonary hypertension in the pathophysiological process of ARDS [16]. KEGG pathways enrichment analysis showed that 33 signaling pathways were significantly enriched in the LPS (ARDS lung injury) group and the DEGs were significantly involved in the chemokine, IL-17, and TNF signaling pathways.

In this study, GSEA showed that both autophagy- and apoptosis-related genes were upregulated in the LPS group (Figures 4(a) and 4(b)), which had significant biological functions. Moreover, signal transducers and activators of transcriptions (STATs) play an important role in this biological process. In normal cells, the activation of STAT3 is tightly controlled to avoid abnormal gene expression [17]. However, the phosphorylation of STAT3 reaches its peak at 15-60 min after stimulation, such as cytokines, activating the STAT3, which plays an important role in cell proliferation, survival, inflammatory responses, invasion, metastasis, and angiogenesis [18]. Activated STAT3 forms a dimer, enters the nucleus, and binds to downstream Cyclin D1, Cyclin B, and cdc2 promoters to initiate transcription and promote the process of the cell cycle, thereby playing an important role in promoting cell proliferation [19]. In addition, it also promotes the survival of injured cells and inhibits apoptosis by regulating the gene expression of anti-apoptotic proteins [20], such as Survivin, Bcl-2, BclxL, and Mcl-1.

PPI network analysis of 130 co-expressed DEGs showed a total of 130 node proteins and 419 interacting edges, with an average node degree of 6.45. This strong interaction network among the DEGs also indicated that the differential proteome might play a biological activity as a whole in the pathogenesis of ARDS lung injury. The further analysis of top 15 key proteins showed that their main biological activities were concentrated on two categories, including inflammatory cytokines, such as STAT3, FCGR1A, and CD14, and chemokines, such as CXCL10 and CXCR1. The qRT-PCR validation study was conducted on the PBMC samples of 20 patients with ARDS. The results showed that the expression of *CYBB*, *CD14*, *CXCL10*, *FCER1G*, *CXCR1*, *FCGR1A*, and *STAT3* was different between the two groups.

The data also showed that blocking the chemokine signal pathways and conditioning the inflammatory cells to lung tissue-specific chemotaxis might alleviate lung injury through biologically targeted treatment [21]. CXCL10, also known as interferon-inducible protein-10 (IP-10), belongs to the CXC chemokine subfamily and is mainly produced by the interferon-*γ*-stimulated monocytes, endothelial cells, and fibroblasts. Binding to its receptor, CXCR3 induces the recruitment of neutrophils, T lymphocytes, mast cells, natural killer cells, etc. [22]. The site of inflammation and plays an important role in the body's immune system. In this study, the expression of CXCL10 and CXCR3 was significantly upregulated in lung tissue of LPS-induced endogenous ARDS rats. CXCL10 promoted the occurrence and development of lung injury by binding to CXCR3 [23]. In addition, in our previous study, it was confirmed that the level of CXCL10 increased significantly in ARDS patients and the enhanced inflammatory response promoted the progression of lung injury [24]. Therefore, it was suggested that the CXCL10/CXCR3 pathway might play an important role in the mechanism of lung injury during endogenous ARDS.

In this study, mRNA-miRNA-lncRNA-circRNA network analysis was performed to obtain the correlation between miRNA and non-coding RNA. The constructed ceRNA network contained a total of 69 nodes and 73 correlation pairs. Differentially expressed miRNAs between ARDS rats and normal rats were screened to identify miRNAs related to ARDS progression. The results showed that the expression of miR-21-3p was significantly up-regulated in ARDS rats. Wang et al. [25] confirmed that the upregulation of miR-21-3p significantly reduced pulmonary oxygenation in a rat model of acute hemorrhagic necrotizing pancreatitis and aggravated pulmonary pathological damage. Furthermore, Xiao et al. [26] reported the upregulation of miR-21-3p expression in lung tissue of adult mouse asthma models, which highly correlated with the level of asthma-promoting Th2 cytokines in mouse bronchoalveolar lavage fluid. In addition, in many studies, it has been confirmed that the expression of miR-21-3p in patients with chronic heart failure and pulmonary infection complications or those with severe acute pancreatitis with lung injury complications was higher than that of patients with simple chronic heart failure or severe acute pancreatitis [27, 28]. This increased expression of miR-21-3p suggested that lung infection or lung injury might lead to the up-regulation of miR-21-3p. All the above studies suggested that miR-21-3p might be significantly related to changes in lung function. In another study [29], it was confirmed that this miRNA was up-regulated in ApoE -/- carotid artery injury mouse models, suggesting its close correlation with vascular intimal injury. In addition, the expression of miR-21-3p was significantly upregulated in hypoxia-induced brain tissue damage and inflammatory factor-induced human aortic endothelial cell injury, and its knockdown alleviated tissue damage by inhibiting inflammatory factors, inflammatory signaling pathways, or cell damage [30, 31]. These studies suggested that miR-21-3p might play an important role in the process of lung injury and vascular disease. It was inferred that the effect of miR-21-3p on ARDS lung injury might be closely related to hypoxia and inflammation-induced lung injury and hyperproliferation, migration, and phenotype conversion of vascular smooth muscles.

Using miRanda, the downstream targets of miR-21-3p were predicted, which showed Camk2g (CaMKII *γ*) as a downstream target. The expression of CaMKII*γ* in normal rats was significantly higher than those in ARDS rats and significantly and negatively correlated with miR-21-3p expression. CaMKII is a multifunctional calcium/calmodulin-dependent serine/threonine protein kinase, which controls a variety of calcium-dependent processes and is widely present in mammalian cells [32]. CaMKII is usually encoded by *α*, *β*, *γ*, and *δ* genes, which plays an important role in maintaining the homeostasis, metabolism, and signal transduction in cells. At present, studies on the correlation between CaMKII and vascular lesions, especially vascular smooth muscle cell (VSMC) proliferation and migration, have been conducted. For example, Nguyen et al. [33] confirmed that, in a VSMC-selective mitochondrial CaMKII knockout mouse model, neointimal hyperplasia was significantly reduced after vascular injury, thereby suggesting that CaMKII expression was closely related to VSMC hyperproliferation and migration.

## 5. Limitations

This study has some limitations. First, we only validated several DEGs of mRNA targets, and lacked validation of differentially expressed lncRNAs and miRNAs. Second, we obtained whole transcriptomic data of the rat ARDS model using high-throughput methods at 36 hours only without dynamic monitoring of the trend in the changes, while more time points need to be evaluated in future studies. Third, in our research, the expression levels of FPR1, CXCR1, FCGR1A, and STAT3 in the ARDs group and the control group showed opposite results in Figures 6(a) and 6(b). We think that it may be due to some differences in gene expression between different species or tissues. And there may be differences in gene expression levels in different stages of the disease, such as the pro-inflammatory stage or the anti-inflammatory stage of the disease; the expression of cytokines may be quite different. At last, the mechanism underlying these findings should be studied in future studies.

## 6. Conclusions

Chemotaxis, migration, and degranulation of inflammatory cells, cytokine immune response, autophagy, and apoptosis have significant biological functions in the occurrence and development of endogenous acute lung injury during ARDS. The camk2g/miR-21-3p/lncRNA/circRNA network, CXCL10/CXCR3, and IL-17 signaling pathways might provide novel insights and targets for further studying the lung injury mechanism and clinical treatment.

## Figures and Tables

**Figure 1:** Pathological changes in lung tissue of two groups of rats: (a) pathological changes in lung tissues of the LPS group, 40×; (b) pathological changes in the lung tissue of the LPS group, 200×; (c) pathological changes in lung tissue of the control group, 40×; and (d) pathological changes in lung tissues of the control group, 200×.

**Figure 2:** mRNA and lncRNA expression abundance Boxplot (a), PCA (b), and sample correlation coefficient matrix heat map (c).

**Figure 3:** Volcano plots of the two sample groups (a-d) and heatmaps of the top 40 DEGs of lncRNAs and mRNAs (e and f).

**Figure 4:** GO/KEGG enrichment analysis of DEGs and GSEA plots of all detected genes. (a-d) Enrichment of gene sets in autophagy, apoptosis, calcium ion pathway, and platelet calcium ion regulation, respectively. (e) Bubble plot showing the distribution of DEGs in three functional groups: molecular function (MF), biological process (BP), and cellular component (CC). (f) Bubble plot showing the distribution of DEGs in Kyoto Encyclopedia of Genes and Genomes (KEGG).

**Figure 5:** (a) Protein-protein interaction (PPI) network. (b) Venn diagram of the two datasets. (c) subnetwork analysis of top 15 hub genes from the PPI network. (d) mRNA-miRNA-lncRNA-circRNA regulatory network diagram.

**Figure 6:** (a) Expression of key genes in rat lung tissue using the whole transcriptome assay. (b) Boxplot, representing the 15 key genes in ARDS patients and healthy controls of GSE32707. (c) Validation of the expression of key genes in ARDS patients and healthy samples using qRT-PCR.

**Table 1:** Primer sequences of the selected genes.

Primer name	Forward primer (5′- >3′)	Reverse primer (5′- >3′)	Primer base pair
HCK	AGGGCTACATCCCAAGCAAC	GGTCTCGCTATCCCGGATCA	152
FGR	GGGCAGCAGACCACTATGG	CCAGGGTTGATGGCCTGAG	106
S100A9	CCACGAGAAGATGCACGA	CCTGGTTGGGTAGAGGCA	185
CYBB	ACCGGGTTTATGATATTCCACCT	GATTTCGACAGACTGGCAAGA	135
SPI1	GCGACCATTACTGGGACTTCC	GGGTATCGAGGACGTGCAT	156
CD14	ACGCCAGAACCTTGTGAGC	GCATGGATCTCCACCTCTACTG	122
CXCL10	GTGGCATTCAAGGAGTACCTC	TGATGGCCTTCGATTCTGGATT	198
FPR1	GTTGACGGTGAGAGGCAT	CGTAAGGGACGACTGGAC	132
FCER1G	TGTTTACACGGGCCTGA	TGAGGGCTGGAAGAACC	128
CSF3R	GCCAGAGGTGCCAACAT	AGTTTCCCAGCCTTGCC	114
CXCR1	AGAAAGAGGGTTTGGAAGC	CAGAGGGGAAGGGCTAA	137
FCGR1A	GCGAAGTGACCCCATACA	TCCACGCATGACACCTC	110
AQP9	GCTGATCGTGGGAGAAAA	TGGAGTCAAAGATGGCAAA	140
RAC2	GCATCTACCCGTTCACTCC	AAGAGCCCCATCCCTGA	107
STAT3	GGACTGAGCATCGAGCA	GCCAGACCCAGAAGGAG	139
GAPDH	CAACAGCCTCAAGATCATCAGCAA	GTCATGAGTCCTTCCACGATACC	105

**Table 2:** GO and KEGG enrichment of DEGs.

Ontology	ID	Description	Gene ratio	Bg ratio	*P* value	*P* adjust	*Q* value
BP	GO:0032496	Response to lipopolysaccharide	67/755	499/17962	2.52e-17	1.27e-13	1.01e-13
BP	GO:0098542	Defense response to other organism	65/755	488/17962	1.16e-16	2.93e-13	2.32e-13
BP	GO:0030595	Leukocyte chemotaxis	40/755	208/17962	4.68e-16	7.87e-13	6.23e-13
BP	GO:0030593	Neutrophil chemotaxis	27/755	96/17962	1.48e-15	1.87e-12	1.48e-12
BP	GO:0019221	Cytokine-mediated signaling pathway	53/755	369/17962	3.73e-15	3.76e-12	2.98e-12
CC	GO:0034702	Ion channel complex	36/769	295/18446	7.88e-09	3.41e-06	3.04e-06
CC	GO:1902495	Transmembrane transporter complex	37/769	315/18446	1.37e-08	3.41e-06	3.04e-06
CC	GO:1990351	Transporter complex	37/769	322/18446	2.47e-08	4.08e-06	3.64e-06
CC	GO:0034703	Cation channel complex	29/769	222/18446	5.07e-08	6.29e-06	5.62e-06
CC	GO:0031012	Extracellular matrix	37/769	362/18446	4.92e-07	4.88e-05	4.36e-05
MF	GO:0005125	Cytokine activity	40/723	177/16882	2.17e-18	1.77e-15	1.56e-15
MF	GO:0008009	Chemokine activity	18/723	37/16882	1.57e-15	6.39e-13	5.62e-13
MF	GO:0030545	Receptor regulator activity	62/723	476/16882	3.92e-15	1.06e-12	9.35e-13
MF	GO:0048018	Receptor ligand activity	58/723	441/16882	2.06e-14	4.20e-12	3.69e-12
MF	GO:0005126	Cytokine receptor binding	42/723	296/16882	7.64e-12	1.24e-09	1.09e-09
KEGG	rno04060	Cytokine-cytokine receptor interaction	56/379	277/9437	1.05e-24	2.98e-22	2.49e-22
KEGG	rno04061	Viral protein interaction with cytokine and cytokine receptor	26/379	86/9437	1.70e-16	2.42e-14	2.02e-14
KEGG	rno04657	IL-17 signaling pathway	24/379	96/9437	2.77e-13	2.63e-11	2.19e-11
KEGG	rno04668	TNF signaling pathway	24/379	116/9437	2.23e-11	1.58e-09	1.32e-09
KEGG	rno04064	NF-kappa B signaling pathway	19/379	106/9437	3.42e-08	1.94e-06	1.62e-06

## Data Availability

The data used to support the findings of this study are uploaded on geodataset, and the BioProject ID: PRJNA875078. All data can be downloaded directly from http://www.ncbi.nlm.nih.gov/bioproject/875078 upon request.

## Abbreviations

ARDS: Acute respiratory distress syndrome
SARS: Severe acute respiratory syndromes
COVID-19: Corona virus disease-19
ICU: Intensive care unit
LPS: Lipopolysaccharide
DEGs: Differentially expressed genes
GO: Gene ontology
KEGG: Kyoto encyclopedia of genes and genomes
qRT-PCR: Real-time quantitative polymerase chain reaction
BPs: Biological processes
CC: Cellular components
MF: Molecular functions
ceRNA: Competing endogenous RNA
PBMCs: Peripheral blood mononuclear cell
GAPDH: Glyceraldehyde-3-phosphate dehydrogenase
GSEA: Gene set enrichment analysis
IL-17: Interleukin-17
TNF: Tumor necrosis factor
NF-*κ*B: Nuclear factor kappa-B
HCK: Hemopoietic cell kinase
FGR: Fetal growth restriction
CYBB: Cytochrome b-245 beta chain
SPI1: Salmonella pathogenicity island 1
CXCL10: Chemokine C-X-C ligand 10
FPR1: Formyl peptide receptor 1
FCER1G: Fc receptor gamma
CSF3R: Colony-stimulating factor receptor
CXCR1: G protein-coupled receptor1
FCGR1A: Fc fragment of IgG receptor 1a
AQP9: Aquaporin 9
RAC2: Rac family small GTPase 2
STAT3: Signal transducer and activator of transcription 3
Camk2g: Calcium ion/calmodulin-dependent protein kinase II gamma
Stx2: Shiga toxin 2
VSMC: Vascular smooth muscle cell.
